The article "Design of Deep Learning Model for Task-Evoked fMRI Data Classification" was published in 2021. Journal: Comput Intell Neurosci.

# Design of Deep Learning Model for Task-Evoked fMRI Data Classification

**DOI:** 10.1155/2021/6660866

**Published:** 2021-08-12

**Authors:** Xiaojie Huang, Jun Xiao, Chao Wu

**Affiliations:** ^1^Polytechnic Institute, Zhejiang University, Hangzhou, China; ^2^College of Computer Science and Technology, Zhejiang University, Hangzhou, China; ^3^School of Public Affairs, Zhejiang University, Hangzhou, China

## Abstract

Machine learning methods have been successfully applied to neuroimaging signals, one of which is to decode specific task states from functional magnetic resonance imaging (fMRI) data. In this paper, we propose a model that simultaneously utilizes characteristics of both spatial and temporal sequential information of fMRI data with deep neural networks to classify the fMRI task states. We designed a convolution network module and a recurrent network module to extract the spatial and temporal features of fMRI data, respectively. In particular, we also add the attention mechanism to the recurrent network module, which more effectively highlights the brain activation state at the moment of reaction. We evaluated the model using task-evoked fMRI data from the Human Connectome Project (HCP) dataset, the classification accuracy got 94.31%, and the experimental results have shown that the model can effectively distinguish the brain states under different task stimuli.

## 1. Introduction

The fMRI data showed which parts of the brain participate in specific psychological processes by detecting the corresponding activation states generated by blood oxygen-dependent dynamic changes that occur in response to neural activities [1]. Decoding and distinguishing different task states from fMRI data is a major research direction at present. Classification of fMRI data is an efficient way to decode the current cognitive state of the brain from subjects, which is of great significance for analyzing the working mechanism of the human mind. This paper aims to classify fMRI signals by establishing a model and classify the different activation states generated by the brain of the subjects under different task stimuli, to study and reveal daily human behaviors and psychological activities more pertinently. In the past few years, machine learning has developed to become a working horse in brain imaging and computational neuroscience, because it helps to mine a large amount of neural data and detect tiny signals from the overwhelming noise floors [2]. The fMRI data classification methods can be roughly divided into two categories: methods based on traditional machine learning and methods based on deep learning.

In traditional machine learning methods, using a general linear model to separate stimulus-induced signals from noise and extracting the features from a specific task are commonly adopted [3]. Under the linear assumption, the linear method significantly reduces the data size to a single voxel or correlation matrix, but this blurs the dynamic and nonlinear characteristics of the blood oxygen-dependent response. The fMRI signals consist of a variety of wave sources, which complicates the analysis of signals related to changes that are truly related to brain activation. Nonhomologous signals are classified by using Independent Component Analysis (ICA) and finding common features in the data [4]. The method of processing and analyzing features based on individual voxels as independent units ignores the correlation between voxels. To add this correlation to improve the understanding of neural signal analysis, multivariate analyses can take advantage of the information contained in activity patterns across space from multiple voxels. Such analyses have the potential to greatly expand the amount of information extracted from fMRI datasets [5]. Traditional machine learning is not entirely reliable and still has some deficiencies, it is mostly a shallow model, its limitation lies in its limited ability to express complex functions with limited samples and computational units, and its generalization ability is limited when dealing with classification problems of high-dimensional data such as functional magnetic resonance imaging. Moreover, it is usually necessary to manually construct features when processing data, which is not only costly but also difficult to describe the rich intrinsic information of data. It may even lead to the discarding of some voxels with weak correlation and fail to make full use of the useful information implied between voxels.

In recent years, deep learning has made many innovative achievements in the field of computer vision; the layers of DNN with nonlinear activation functions can learn more complex output functions than traditional machine learning methods [6]. The deep neural network algorithm is also applied to the field of neural images. DNN can extract advanced features from the original input data, and the facts prove that these features have better representation ability than manual features [7]. Deep Belief Network (DBN) uses the low-dimensional representation of fMRI data to decode the brain. This method flattens the three-dimensional image into a one-dimensional vector as the feature of learning DBN, which makes the three-dimensional fMRI data lose the spatial structure information [8]. The 2D convolution is widely used in image classification; Hu proposed M2D CNN, a novel multichannel 2D CNN model, to classify 3D fMRI data. The model uses sliced 2D fMRI data as input and integrates multichannel information learned from 2D CNN networks [9]. However, according to the characteristics of functional data, this is four-dimensional data, containing most of the temporal and spatial information of brain activity [10]. At present, most feature methods do not directly analyze four-dimensional fMRI data, so these methods more or less lose the temporal and spatial information in fMRI data. A deep 3D convolution neural network can effectively and reliably perform the classification and identification tasks of functional networks. At the same time, it can achieve a good training effect even if the data contain high error marks [11]. The deep learning method is good at extracting information from high-dimensional data space and can learn highly complex and abstract features from data. Therefore, it is a more robust method than traditional machine learning, and the convolution network has a strong feature extraction ability in spatial information processing. 3D convolution model is used to model fMRI data, which can distinguish brain activation states under different task stimuli [12]. According to the characteristic that fMRI data contain time-series information, the LSTM network can be used to distinguish different task states on fMRI data, which can obtain better brain decoding performance than traditional methods [13]. For the deep learning model, the convolutional neural network has a sufficient ability to extract local features. However, fMRI data are inherently four-dimensional imaging data with time series. Most of the current methods only focus on spatial features and ignore the temporal sequential changes of voxels. It shows that both temporal and spatial information are critical in fMRI data, so it is of great research significance to design a model that can analyze both sequential and spatial information on fMRI data.

Therefore, we propose a deep network based on the spatiotemporal information feature of four-dimensional fMRI data. We use the convolution network to extract spatial features and the recurrent network to extract temporal sequential features. Finally, the feature extracted above is sent to a classifier for classification. To sum up, our contributions are as follows:

1. We add time distribution processing to each convolution layer and aggregation layer so that the convolution network retains the time information of the original data. And we set a full convolution in the last layer of the convolution network, which effectively reduces the training parameters and slows down the occurrence of overfitting.
2. The bidirectional LSTM layer is added to process data timing information, and we use the attention mechanism to improve the model's capture of important information in time sequences.

## 2. Materials and Methods

### 2.1. Data Introduction

The dataset we used is Wu-Minn Human Connectome Project (HCP) [14, 15], which is a large public dataset of fMRI data. It includes several classes of fMRI data such as structural MRI data, resting fMRI data, and task-evoked fMRI data, among which task-evoked fMRI dataset contains seven different task-evoked data: Emotion, Gambling, Language, Motor, Relational, Social, and Working Memory. During the task, the subject's brain will be continuously scanned by the magnetic resonance data acquisition instrument, and at the same time, the subject will receive video prompts at different task stages to ask them to perform corresponding actions. The Emotion task requires the subject to choose which of the two facial expressions with the label “fear” or graphic shapes with the label “neur” presented at the bottom of the screen matches the facial expression or graphic shape at the top of the screen. Gambling task requires the subjects to participate in the card guessing game and determines the brain reaction when the subjects lose with the label “lose” or win with the label “win” by guessing the numbers on the mysterious card. The Language task requires the subjects to listen to a short story adapted from Aesop's fable with the label “Story” or a simple math problem with the label “Math” and then choose the theme that matches the story or choose the answer corresponding to the topic. For the Motor task, the subjects will receive visual prompts to ask them to perform corresponding actions, including hitting their left hand with the label “Left Hand” or right hand with the label “Right Hand,” squeezing their left foot with the label “Left Foot” or right foot with label the “right root,” or moving their tongue with the label “Tongue.” The Relational task judges whether objects are related to the label “relation” or matched with the label “match” by showing short video clips to subjects. For Social tasks, the subjects will watch a short video and then judge whether the objects in the video have mental interaction with the label “mental” or no interaction with the label “rnd.” For the Working Memory task, the subjects were presented with an experiment consisting of pictures of places with the label “places,” tools with the label “tools,” faces with the label “faces,” and body parts with the label “body” and then recorded the changes of the brain under four types of stimuli. According to the characteristics of fMRI data collection, the subjects will participate in each task, each task is composed of several different subtasks, each subtask will be executed several times, and each task will last for several seconds. We only selected one subtask as the sample of each task, as shown in Table 1.

### 2.2. Data Processing

The spatial dimension of HCP data is 91 × 109 × 91x frames. We cut out some useless information such as black borders in the space to get fMRI data with a dimension of 78 × 93 × 76x frames. In addition, to satisfy the condition of the hemodynamic response function, we not only considered the duration of the whole task block but also covered the time of 8 s after the task block for each sample. Then, according to the duration of the whole task and the total number of frames, the sampling repetition time of the task state fMRI data of HCP can be calculated to be 0.72, and the selected subtask block segmentation method is shown in formula

(1) $$\begin{array}{c} \text{TF}=\frac{\left(\text{TD}+8\right)}{0.72}\text{.} \end{array}$$

Here, TF represents the total number of task sample frames and TD represents the task duration. After obtaining the total number of frames of subtask, it is only necessary to calculate the position of frames corresponding to the start time and then extract subtask samples with corresponding frames from the whole sample according to the frames corresponding to the start time and the frames corresponding to the end of the task. The number of frames and samples corresponding to a single subject in seven tasks is shown in Table 2.

Because the durations of different subtasks are not the same and the frames corresponding to the extracted task samples are not the same, it is necessary to unify the frames of different task samples before taking the samples as the input of the model. In the experiment, 21 consecutive frames in subtasks are selected as separate samples. When the data amount of depth model is small, the model is prone to overfitting, which will show a good effect on the training set and poor effect on the test set. At this time, it is necessary to increase the amount of data in the training set to improve the performance of the model. However, the dataset of HCP has been spatially aligned by the standard MNI152 template, so it can only be enhanced in the time dimension. First, randomly collect 21 consecutive brain images in a single task block as new samples, and then repeat them many times. The number of repetitions needs to be determined according to the number of task blocks in Table 3. Because different tasks are executed at different times, to ensure that the number of samples of each task in the training set is the same, the data imbalance will cause the model to be biased towards the prediction of a certain task. Therefore, we need to carry out balanced sampling here, so that the number of task blocks of each subject after enhancement reaches 12 samples.

According to the characteristics of blood flow in fMRI, when there is a blood oxygen reaction in images, there will be obvious differences between frames. The absolute value of the brightness difference between the two frames can be obtained by subtracting two frames to judge whether there is a blood oxygen reaction in the brain area. In the experiment, 21 frames of samples were extracted and then subjected to the interframe difference method to obtain 20 frames of samples. Data normalization is a basic work of data mining. In the experiment, we normalized the 3D brain image in the data time dimension, and the processing method is shown in formula (2), in which *X*_*i*_ represents the brain image of the *i*_th_ frame and *X*^*∗*^ represents the normalized brain image, which is obtained by dividing each frame of brain image by the frame with the largest brain image value in the current sample:

(2) $$\begin{array}{c} X_{i}^{*}=\frac{X_{i}}{\max\left(X_{1},X_{2},\ldots ,X_{20}\right)}. \end{array}$$

The above is the data prepossessing. In addition, we need to divide the whole dataset into the training set, validation set, and test set according to the number of subjects for training and verification. The division ratio is 80% as the training set, 10% as the validation set, and 10% as the test set. The whole data processing flow is shown in Figure 1.

### 2.3. Model Overview

We input the fMRI data into the model as input *X* [*t*, *x*, *y*, *z*, *c*]. Firstly, the convolution network extracted spatial features and effectively reduced the size of the fMRI data dimension. The operation of the convolution structure can be expressed as follows:

(3) $$\begin{array}{c} X_{\text{cnn}}=\text{cnn}\left(X\right). \end{array}$$

The output *X*_cnn_ from the convolution network is reshaped to *X*_cnn_ [*t*, *h*] and then input into the RNN network, and the timing characteristics are extracted through the RNN network. The processing of the RNN network can be expressed as follows:

(4) $$\begin{array}{c} X_{\text{rnn}}=\text{rnn}\left(X_{\text{cnn}}\right). \end{array}$$

Finally, the output of the RNN network is input into the classification network as input *X*_rnn_ [*h*] to obtain the final prediction result, which can be expressed in the following form as a whole:

(5) $$\begin{array}{c} X_{\text{pred}}=\text{classifier}\left(X_{\text{rnn}}\right). \end{array}$$

The prediction results correspond to our classification target.  Figure 2 shows the overview of our model. Next, we will describe the network separately in this overview in detail.

### 2.4. CNN Architecture

Firstly, here is the CNN network [16]. Two-dimensional convolution extracts the features of two-dimensional natural images, while three-dimensional convolution is used to extract the features of three-dimensional brain imaging data. However, fMRI data contain time series, so we added a trick in the forward propagation of data, that is, making the same convolution kernel to convolution operation at each scanning point to maintain time-series information. The structure is shown in Figure 3.

The CNN network consists of four convolution blocks, each of which includes a convolution layer, a BatchNorm layer, and a ReLU activation layer. And the parameters are set as shown in Table 2.

The data are input into the convolution layer through feature extraction of the convolution layer:

(6) $$\begin{array}{c} x_{j}^{l}=\sum_{i\in M}x_{i}^{l-1}*k_{j}^{l}+b^{l}, \end{array}$$

where *l* represents the *l*_th_ convolution block, *M* represents the set of feature maps, *x*_*i*_ represents the *i*_th_ input feature map, *k*_*j*_ represents the *j*_th_ convolution kernel, *x*_*j*_ represents the *j*_th_ output feature map, and *b* is the bias. The output of each convolution layer is batch normalized by BatchNorm layer [17]; BatchNorm forcibly pulls the distribution of the input value of any neuron in each layer of the neural network back to the standard normal distribution with a mean value of 0 and a variance of 1 through a specific normalization method:

(7) $$\begin{array}{c} x_{bn}=\gamma \cdot \frac{x_{j}^{l}-\mu }{\sqrt{\sigma^{2}+\varepsilon }}+\beta . \end{array}$$

After the batch normalization operation, a nonlinear transformation is performed by the ReLU activation function [18]:

(8) $$\begin{array}{c} x_{\text{conv}}^{l}=\text{Relu}\left(x_{bn}\right). \end{array}$$

We adopted a stride of two in the first three convolutional layers to compress the size of data instead of the pooling layer, which can reduce the dimension to some extent and reduce the amount of computation. And the last convolutional block is a fully convolutional layer. The dimension of the feature map generated by each layer of the convolution block will be reduced. The first three layers are commonly used in convolution networks. First, we used a large receptive field to extract features; then, we used two conventional receptive fields to extract features. In the last convolution block, we used the full convolution which could be treated as a fully connected layer so that the kernel of this layer can cover the information of the last feature map, and the final output shape is [20, 1, 1, 1, 64].

### 2.5. RNN Architecture

Secondly, we reshape the feature map from the last convolution block to the shape of [20, 64]; then, we used the RNN network to extract the temporal sequential feature. The structure of the RNN is shown in Figure 4.

The structure of RNN network includes two hidden LSTM layers [19]: the LSTM layers are used to extract information on the temporal dependency for each time point and the information representation extracted in each LSTM layer is calculated as

(9) $$\begin{array}{c} f_{t}^{l}=\sigma \left(W_{f}^{l}\cdot \left[h_{t-1}^{l},x_{t}^{l}\right]+b_{f}^{l}\right),\\ i_{t}^{l}=\sigma \left(W_{i}^{l}\cdot \left[h_{t-1}^{l},x_{t}^{l}\right]+b_{f}^{l}\right),\\ {\tilde{C}}_{t}^{l}=\tanh\left(W_{C}^{l}\cdot \left[h_{t-1}^{l},x_{t}^{l}\right]+b_{c}^{l}\right),\\ C_{t}^{l}=f_{t}^{l}*C_{t-1}^{l}+i_{t}^{l}*{\tilde{C}}_{t}^{l},\\ h_{t}^{l}=\sigma \left(W_{o}^{l}\cdot \left[h_{t-1}^{l},x_{t}^{l}\right]+b_{o}^{l}\right)*\;\tanh\left(C_{t}^{l}\right), \end{array}$$

where *f*, *i*, *c*, *h*, and *x* denote the output of forget gate, input gate, cell state, hidden state, and the input feature vector of the *l*_th_ LSTM layer at the *t*_th_ time point, respectively, and *σ* denotes the sigmoid function. The RNN network consists of two LSTM layers, and each LSTM layer is followed by a dropout layer [20]. Dropout layer will randomly set some neurons invisible with a probability of 0.2, and the input and output neurons will remain unchanged. This two LSTM layers are with opposite directions, so that it is called bidirectional LSTM, and each layer is with 64 units. It involves duplicating the first recurrent layer in the network so that there are now two layers side by side, then providing the input sequence as-is as input to the first layer, and providing a reversed copy of the input sequence to the second. Finally, we merge these two LSTM layers with opposite directions by concatenating them. The input features to the LSTM layer are the feature vector derived from the CNN network.

### 2.6. Attention Mechanism

The essence of the attention mechanism is to locate interesting information and suppress useless information [21]. It is to calculate the weight of each time series first and then take the weighted sum of all time-series vectors as feature vectors. The specific processing process of attention has the following formula:

(10) $$\begin{array}{c} c_{i}=\sum_{i=1}^{T_{x}}w_{j}h_{j}, \end{array}$$

and *w*_*j*_ is

(11) $$\begin{array}{c} w_{j}=\frac{\exp\left(h_{j}\right)}{\sum_{k=1}^{T_{x}}\exp\left(h_{k}\right)}. \end{array}$$

In the above formula, *T*_*x*_ is the total time steps, and *h*_*j*_ is the output of the *j*_th_ time of the previous hidden layer and in our model here is the output of the LSTM layer. It can be found that the model for calculating *c*_*i*_ is a linear summation model, and *w*_*i*_ is actually the weighted average of the outputs of hidden layers at each time in the previous hidden layer. After adding the attention mechanism to the RNN module, the attention mechanism structure is shown in Figure 5.

### 2.7. Classifier Architecture

Finally, we used the classification network to obtain the final classification results; the structure of the classification network is shown in Figure 6.

The structure of the classifier includes two fully connected layers; the dense layers are used to learn a mapping between the learned feature representation. The first dense layer with 64 hidden units and the last fully connected layer with softmax activation function are adopted for the classified 7 task states as

(12) $$\begin{array}{c} s=\text{softmax}\left(W_{s}\cdot h+b_{s}\right), \end{array}$$

where *s* is the prediction vector with the number of task probability predictions and *h* is the hidden state output of the first dense layer. These are the details of the model. Parameters *W* and *b* will be continuously optimized during the training process of the experiment. Then, we use the output of the model and the real label to input into our loss function, which is a commonly used cross-entropy loss function to calculate the loss value; then, we use the backpropagation method to update the parameters of the model according to this loss value:

(13) $$\begin{array}{c} p_{i}=\text{softmax}\left({\text{logits}}_{i}\right)=\frac{e^{{\text{logits}}_{ij}}}{\sum_{j=0}^{\text{numclasses}-1}e^{{\text{logits}}_{ij}}},\\ {\text{loss}}_{i}=-\sum_{j=0}^{\text{numclasses}-1}y_{ij}*\;\ln\;p_{ij}, \end{array}$$

where *y* represents the true label value, logits represents the output of the model, and a probability vector *p* is obtained by the activation function of softmax with the input of logits; then, the loss value is calculated by the cross-entropy function.

### 2.8. Comparison Models

Given the above model we designed, we also use the following models as benchmarks for comparison of classification performance when given the same input data and output categories.

#### 2.8.1. MLP

The structure of the MLP model is described in Section 2.7. The input is four-dimensional fMRI data (20 × 78 × 93 × 76), so firstly, the input should be processed, and the time dimension of fMRI data should be averaged to transform the four-dimensional fMRI data into one frame of average three-dimensional brain image data (78 × 93 × 76). Then, all voxel points of the three-dimensional brain imaging sample are flattened into one-dimensional vectors with 551,304 features, which are input into a one-dimensional vector containing a fully connected layer and one-dimensional vectors.

#### 2.8.2. BiLSTM

The structure of the BiLSTM model is described in Section 2.5. In this model, only the time information of fMRI data is considered, and the three-dimensional brain image information is directly flattened into one-dimensional vector features. Firstly, four-dimensional fMRI data (20 × 78 × 93 × 76) are transformed into feature vectors (20 × 551304) containing time series and then input into the bidirectional long-term and short-term memory network for extracting the time-series features from the data. The hidden units in each layer of the bidirectional LSTM layer are 64, the value of the dropout layer is 0.2, and then an attention mechanism is connected to the process and assigns weights to each time point. Then, it is input into the fully connected layer with 64 nodes for further processing. Finally, the probability value of each category is calculated by the softmax function of the output layer for classification.

#### 2.8.3. M2D CNN

In the multichannel 2D CNN model [9], averaging is also carried out on the time dimension of fMRI data, the four-dimensional fMRI data (20 × 78 × 93 × 76) are transformed into three-dimensional brain image data (78 × 93 × 76), and then the third dimension of the three-dimensional brain image is input into the two-dimensional convolution network model as a channel, which includes a combination of two-dimensional convolution layers and pooling layers, a fully connected layer, and an output layer.

#### 2.8.4. 3D CNN

The structure of the BiLSTM model is described in Section 2.4. The input format of the model is [batch size, 78, 93, 76, 1]. Firstly, the four-dimensional fMRI data (20 × 78 × 93 × 76) are converted into three-dimensional single-channel brain image data (78 × 93 × 76 × 1), and then single-channel gray-scale three-dimensional brain image samples are input into the three-dimensional convolution network model. The network contains four layers of convolution, and the first three layers are the combination of the convolution layer and the pooling layer. It is used to extract the spatial features of 3D images, which are output by the fourth layer and full convolution, flattened, and input into the full connection layer for further study, and finally, the probability values of each category are calculated by the softmax function of the output layer for classification.

## 3. Experiments

### 3.1. Data Processing

In the experiment, the whole dataset is divided into 10 parts according to the number of subjects. In each experimental training model, 80% was randomly selected as the training set, the remaining 10% as the validation set, and 10% as the test set.

### 3.2. Training

In the experiment, the training models are implemented with the TensorFlow [22] deep learning framework, and Adam is used as the model optimization method. The initial learning rate is set to 0.001, the data matrix of the input model is [20, 78, 93, 76, 1] (time, *x*, *y*, *z*, *c*), and eight samples are input into the model at a time. Because the convolution layer does not process the timing information, the layer wrapper time distributed in Keras is needed to encapsulate the convolution layer, so that the convolution layer maintains the timing information and only extracts the features of the last four dimensions of the data. When the change of loss tends to be flat during the training process or the accuracy of the model on the validation set is not rising, we think that the model has converged; then, we stop training and save the parameters with better results in the model training. The training process is shown in Figure 7.

### 3.3. Validation

After the model trains the whole training set, it will use the verification set to test the performance of the trained model. And the model that performed best will be saved. The results are shown in Figure 8, which shows the performance of the trained model on the seven tasks of the verification set.

### 3.4. Compare the Experimental Test Results

Under the same experimental conditions, we use the following current methods introduced in Section 2.8 to compare the classification performance with our model, and according to the data processing method in Section 3.1, under the condition that other experimental conditions are consistent except for different datasets, we conducted a 10-fold cross-validation test on each model and took the average of the results of 10 models on the test set as the final model test performance result. And the result is shown in Table 4.

Under the same experimental parameter configuration of each model, the total number of model parameters, the number of parameters that the model participates in training, and the number of nodes connected to the full connection layer in the model are shown in Table 5.

Table 4 shows the performance of each model in classification accuracy, precision rate, recall rate, and F1 value. Table 5 illustrates the size of each model and the dimension of the feature vector extracted from the data. The first is the BiLSTM model, which is characterized by processing only the temporal features of fMRI data, while the spatial features are directly flattened into the input model. Due to the characteristics of the recurrent network, the model parameters increase sharply, which easily leads to an overfitting phenomenon under certain data samples. Therefore, the BiLSTM model's performance representation is the worst with only 44.95% classification accuracy. Secondly, the MLP model with the second largest number of parameters does not consider the temporal characteristics of fMRI and the spatial characteristics of data. It adopts the method of violent dimension reduction, taking the average value of the temporal dimension and flattening it directly in space, which directly loses some characteristics of fMRI data, and the number of nodes input into the full connection layer is also the largest, which leads to a sharp increase in the number of model parameters and is also easy to produce overfitting, so the final classification accuracy is only 82.41%. Next, there are two convolutional neural network models, 3D CNN model and M2D CNN model, with a classification accuracy of 89.62% and 87.85%, respectively. What they have in common is that they only extract spatial features from the input data, which is indeed improved compared with the MLP model but does not consider the time-series characteristics of fMRI. One of the highlights of the 3D CNN model is the addition of the full convolution layer in the last layer of the convolutional network, which makes the parameters of nodes input into all connections change after the image passes through the convolutional network. The model designed in this paper comprehensively considers the advantages and disadvantages of the above models. It not only designs the convolution network for the spatial characteristics of fMRI data but also designs the recurrent network for the time-series characteristics of fMRI data. Finally, the extracted feature vector has only 128 feature values, which are then input into the MLP classification module, and the final classification effect can reach 94.31%. Among the above models, our model performs better than other models in terms of classification accuracy, precision, recall, and F1 value. The results show that the model designed in this paper fully considers the temporal and spatial characteristics of fMRI data and can show the best results under the classification of seven tasks.

## 4. Conclusions

In recent years, modeling and analyzing fMRI data by deep learning has become a hot research direction in the field of brain imaging data analysis. However, because of the high dimension and small sample size of fMRI data, it brings great challenges to modeling and analyzing fMRI data by deep learning.

In this paper, by analyzing the existing problems of several deep learning methods in modeling and analyzing fMRI data and fully considering the temporal and spatial characteristics of fMRI data, we proposed a convolutional recurrent neural network model which can deal with both spatial and temporal features. In this model, the designed convolution network module is used to process the three-dimensional spatial information behind fMRI data, the high-dimensional spatial information is transformed into low-dimensional vectors through feature extraction, and then the information of the designed cyclic neural network in time-series dimension is used to extract feature. In this paper, the model we proposed is used for classification experiments on the open dataset of task fMRI and compared with other deep learning methods. Experimental results show that the CRNN model designed in this paper makes full use of the spatiotemporal features of fMRI data and can achieve an average accuracy of 94.31%, which is superior to other comparative deep learning methods.

In general, the method we proposed in this paper can directly extract task-related information from the four-dimensional fMRI time-series data and can classify seven typical task stimuli.

## Figures and Tables

**Figure 1:** Data processing.

**Figure 2:** Overview of our model.

**Figure 3:** The CNN architecture.

**Figure 4:** The RNN architecture.

**Figure 5:** Attention mechanism.

**Figure 6:** The classifier architecture.

**Figure 7:** Workflow of model training.

**Figure 8:** Confusion matrix on validation set.

**Table 1:** Details of seven tasks.

Task	Task duration (min)	Task frames	Selected condition	Condition duration (s)
Emotion	2 : 16	176	Fear	18
Gambling	3 : 12	253	Loss	28
Language	3 : 57	316	Story	24
Motor	3 : 34	284	Left hand	12
Relational	2 : 56	232	Relation	16
Social	3 : 27	274	Mental	23
WM	5 : 01	405	2bk_places	27.5

**Table 2:** Frame number and block number of seven subtasks.

Task	Fear	Loss	Story	Left hand	Relation	Mental	2bk_places
Frames	36	50	44	28	33	43	49
Block	2	2	4	2	3	2	1

**Table 3:** Parameter setting of convolution layer.

Layer	Kernel size	Channels	Steps
Conv1	7 × 7 × 7	32	2
Conv2	3 × 3 × 3	64	2
Conv3	3 × 3 × 3	64	2
Conv4	8 × 10 × 8	64	1

**Table 4:** Comparison results of classification effects of various models.

Model	Accuracy	Precision	Recall	*F*1 score
MLP	82.41% ± 1.06%	82.62% ± 1.07%	80.37% ± 1.17%	80.89% ± 1.18%
BiLSTM	44.95% ± 2.46%	38.11% ± 2.28%	37.90% ± 2.65%	37.12% ± 2.05%
M2D CNN	87.85% ± 1.07%	87.90% ± 1.11%	86.53% ± 1.21%	87.12% ± 1.13%
3D CNN	89.62% ± 1.17%	89.65% ± 0.97%	90.02% ± 0.89%	89.76% ± 0.94%
**Ours**	**94.31%** **±** **1.39%**	**93.92%** **±** **1.27%**	**95.24%** **±** **1.43%**	**94.48%** **±** **1.28%**

**Table 5:** Number of model parameters.

Model	Total parameters	Training parameters	Unit number input into dense layer
MLP	35,283,975	35,283,975	551,304
BiLSTM	282,317,959	282,317,959	128
M2D CNN	1,565,623	1,565,271	12,096
3D CNN	1,988,935	1,988,487	64
Ours	2,882,503	2,882,055	128

## Data Availability

The task-evoked fMRI dataset analyzed during this study is available in the Human Connectome Project repository (http://www.humanconnectome.org/).
